# Marine-Derived Piericidin Diglycoside S18 Alleviates Inflammatory Responses in the Aortic Valve via Interaction with Interleukin 37

This article has been retracted.

**DOI:** 10.1155/2022/6776050

**Published:** 2022-08-17

**Authors:** Shunyi Li, Jianglian She, Jingxin Zeng, Kaiji Xie, Zichao Luo, Shuwen Su, Jun Chen, Gaopeng Xian, Zhendong Cheng, Jing Zhao, Shaoping Li, Xingbo Xu, Dingli Xu, Lan Tang, Xuefeng Zhou, Qingchun Zeng

**Affiliations:** ^1^State Key Laboratory of Organ Failure Research, Department of Cardiology, Nanfang Hospital, Southern Medical University, Guangzhou 510515, China; ^2^CAS Key Laboratory of Tropical Marine Bio-resources and Ecology, Guangdong Key Laboratory of Marine Materia Medica, South China Sea Institute of Oceanology, Chinese Academy of Sciences, Guangzhou 510301, China; ^3^NMPA Key Laboratory for Research and Evaluation of Drug Metabolism, Guangdong Provincial Key Laboratory of New Drug Screening, School of Pharmaceutical Sciences, Southern Medical University, Guangzhou 510515, China; ^4^Guangdong Provincial Key Laboratory of Shock and Microcirculation, Southern Medical University, Guangzhou 510515, China; ^5^Bioland Laboratory (Guangzhou Regenerative Medicine and Health Guangdong Laboratory), Guangzhou 510005, China; ^6^State Key Laboratory of Quality Research in Chinese Medicine, Institute of Chinese Medical Sciences, University of Macau, Macau, China; ^7^Department of Cardiology and Pneumology, University Medical Center of Göttingen, Georg-August-University, Göttingen, Germany

## Abstract

Calcific aortic valve disease (CAVD) is a valvular disease frequently in the elderly individuals that can lead to the valve dysfunction. Osteoblastic differentiation of human aortic valve interstitial cells (HAVICs) induced by inflammation play a crucial role in CAVD pathophysiological processes. To date, no effective drugs for CAVD have been established, and new agents are urgently needed. Piericidin glycosides, obtained from a marine-derived *Streptomyces* strain, were revealed to have regulatory effects on mitochondria in previous studies. Here, we discovered that 13-hydroxypiericidin A 10-*O*-*α*-D-glucose (1→6)-*β*-D-glucoside (S18), a specific piericidin diglycoside, suppresses lipopolysaccharide- (LPS) induced inflammatory responses of HAVICs by alleviating mitochondrial stress in an interleukin (IL)-37-dependent manner. Knockdown of IL-37 by siRNA not only exaggerated LPS-induced HAVIC inflammation and mitochondrial stress but also abrogated the anti-inflammatory effect of S18 on HAVICs. Moreover, S18 alleviated aortic valve lesions in IL-37 transgenic mice of CAVD model. Microscale thermophoresis (MST) and docking analysis of five piericidin analogues suggested that diglycosides, but not monoglycosides, exert obvious IL-37-binding activity. These results indicate that S18 directly binds to IL-37 to alleviate inflammatory responses in HAVICs and aortic valve lesions in mice. Piericidin diglycoside S18 is a potential therapeutic agent to prevent the development of CAVD.

## 1. Introduction

Calcific aortic valve disease (CAVD) is the leading cause of cardiac valvular disorder in developed countries, with the estimated prevalence of 12.6 million cases and more than 2% of the population over 75 years old in 2017 [1]. Calcific aortic valvular, implicated as valvular stenosis, results in progressive left ventricular hypertrophy or obstruction and ultimately ischaemic injury to the heart [2, 3]. However, there is no effective pharmacological treatment to delay CAVD progression other than valve replacement with a mechanical or bioprosthetic valve for late-stage patients with CAVD. Thus, more effective anti-CAVD agents are urgently needed to improve clinical outcomes and to decrease the need for valve replacement in patients.

The pathogenesis of CAVD is complex and multifactorial, with spatiotemporal heterogeneity. Lipoprotein deposition, haemodynamic stress, inflammation, and immune reactions are implicated in the initial and propagated period of CAVD [4]. It is well established from a variety of studies that the inflammation in valve is a characteristic hallmark in the progression of CAVD [5–9]. In previous searches on Meng et al. lipopolysaccharide (LPS), a Toll-like receptor 4 (TLR4) agonist, was found to be an important proinflammatory factor in human aortic valve interstitial cells (HAVICs) and resulted in activation of NF-*κ*B signal pathway and subsequent induction of inflammation in HAVICs [10, 11]. Thus, these findings related to the proinflammatory signal pathway responsible for the anti-inflammatory mechanism in CAVD provide significant insights for the development of therapies.

Increasing evidence suggests that reactive oxygen species (ROS) are overproduced, and antioxidant levels are decreased both in animal models of CAVD and in the calcified aortic valve of patients with CAVD [12, 13]. Mitochondria are the main sources of intracellular ROS, the overproduction of which is responsible for multiple cellular processes involved in cardiovascular diseases, including inflammation, apoptosis, and ossification [14]. Furthermore, the alerts of mitochondria masses and mitochondrial dysfunction result in ROS overexpression to trigger oxidative stress and inflammation [15]. Valerio et al. found that the GSSG-GSH ratio was higher in CAVD patients, which suggests oxidative stress may play a vital role in the development of CAVD [16]. Our previous studies also found that mitochondrial stress is activated in calcified aortic valve and inhibition of mitochondrial stress with N-acetyl-L-cysteine (NAC) treatment attenuates osteogenic responses in HAVICs. In addition, the NF-*κ*B p65 phosphorylation induced by mitochondrial stress is attenuated by NAC treatment [17]. These results indicate that mitochondrial quality control has a prominent effect on maintaining normal aortic valve function. However, the underlying mechanism of mitochondrial stress in HAVICs remains elusive.

Interleukin (IL)-37, a member of the IL-1 family, is known to inhibit innate and acquired immune responses [18]. IL-37 is known to be expressed in human heamatopoietic cells, epithelial cells, breast carcinoma cells, HAVICs, and other cells [18, 19]. Previous research has established that IL-37 has powerful protective effects on inflammatory diseases, autoimmune diseases, and cancers [18, 20, 21]. Additionally, intracellular IL-37 modulates adaptive antitumour immunity through multiple signal pathways, such as the NF-*κ*B pathway, and subsequently suppresses tumour growth [20]. Our previous studies have revealed that IL-37 suppresses LPS-induced inflammatory and osteogenic responses in HAVICs [22]. Thus, IL-37 plays a vital role in the pathobiological process associated with CAVD. Specifically, our data revealed that the expression of IL-37 is decreased in calcified aortic valve compared with those from patients with non-CAVD. These findings suggest that the discovery of anti-inflammatory agents interacting with IL-37 provides an up-to-date strategy for the prevention of CAVD.

Marine-derived microorganisms have an unrivalled potential for drug development and the production of highly potent natural compounds. The piericidin family is an important kind of active microbial metabolite that features a 4-pyridinol core linked with a methylated polyketide side chain [23]. Accumulating evidence suggests that natural piericidins obtained from marine-derived *Streptomyces* have received considerable attention in recent years because of their important medicinal activities [23, 24]. Our group has previously obtained 43 natural piericidins from two strains of marine-derived *Streptomyces*, including 29 new compounds [25–27], and found that the main piericidin metabolites, including piericidin A (PA) and glucopiericidin A (GPA), have the potential to be developed as potential antirenal carcinoma drugs. Mechanistic studies have shown that these piericidins, whether aglycones or glycosides, could reduce ROS levels and regulate oxidative stress, as inhibitors of mitochondrial respiratory chain complex I. Piericidins can inhibit NF-*κ*B activation by forcing the antioxidative protein peroxiredoxin 1 (PRDX1) into the nucleus [25]. The pharmaceutical potential of natural piericidins, especially the antioxidant and anti-inflammatory effects of special glycosides, is still worth further study. In our research, to discover new agents with anti-inflammatory and mitochondrial regulatory effects, the piericidin glycoside GPA and a special piericidin diglycoside, 13-hydroxypiericidin A 10-*O*-*α*-D-glucose (1→6)-*β*-D-glucoside (S18), were screened and studied. The piericidin diglycoside S18 showed potent anti-inflammatory effects in HAVICs. The potential ability of S18 to act as an anti-CAVD agent is worthy of further study. Here, we investigated the effect of piericidin diglycoside S18 in the development of CAVD in vivo and in vitro. A novel anti-CAVD candidate was observed and confirmed in the present study.

## 2. Methods and Materials

### 2.1. Fermentation and Isolation of S18 and GPA

The strain *Streptomyces psammoticus* SCSIO NS126, derived from a mangrove sediment sample collected from the Pearl River estuary of the South China Sea, was fermented in a volume of 100 L, according to a previously described method [25]. The culture broth was extracted with ethyl acetate three times and then concentrated under a vacuum. The extract (75.0 g) underwent chromatography on silica gel to give eight fractions (Frs. 1~8). With the guidance of high-performance liquid chromatography (HPLC) analysis, Frs. 7 was purified with silica gel again to give six subfractions (Frs. 7-1~7-6). Frs. 7-2 was purified by semipreparative HPLC to obtain compound GPA (358 mg), while S18 (58 mg) was obtained and purified by repeated semipreparative HPLC isolation. The obtained compound was determined to be ≥95% purity by analytical HPLC. The structures of the obtained compounds were determined to be GPA and S18 by comparison of high-resolution mass spectrometry (HRMS) and nuclear magnetic resonance (NMR) data (Figures S1-S6) with the literature data [25]. The compounds were stored at -20°C until use and dissolved in DMSO to a stock concentration of 10 mM.

### 2.2. Human Aortic Valves

Human calcified aortic valves were collected from five patients with CAVD who underwent aortic valve replacement in 2020-2021. The clinical features of patients are shown in Supplementary Table S1. Control noncalcified aortic valves were intraoperatively collected from four patients who underwent aortic valve replacement due to acute aortic dissections. The exclusion criteria included infective endocarditis, congenital valve disease, and rheumatic heart disease. CAVD was diagnosed when the leaflet thickness was ≥3 mm, the peak AV velocity was ≥1.5 m/s, and there was increased echogenicity (aortic root echogenicity was the control) [28]. Written informed consent was obtained from all patients in this study. The protocol of this study was conducted in accordance with the Declaration of Helsinki and was approved by the Nanfang Hospital, Southern Medical University.

### 2.3. Cell Culture and Treatment

HAVICs were isolated and cultured as previously reported [17]. In brief, valve leaflets were subjected to digestion with collagenase, and cells were collected by centrifugation. The cells were cultured in M199 growth medium (Gibco, C11150500BT) containing penicillin G, streptomycin, and 10% fetal bovine serum. Cells from passages 3-6 that reached 80-90% confluence were used for this study.

To determine the influence of S18 on the inflammatory responses in LPS-stimulated HAVICs, HAVICs were treated with LPS (200 ng/mL, Sigma, L4391) in the absence or presence of S18 (0.5 *μ*M) for 24 hours.

To evaluate the role of NF-*κ*B in the suppression of HAVIC inflammation by S18, HAVICs were treated with LPS (200 ng/mL) in the absence or presence of S18 (0.5 *μ*M) for 4 hours.

To determine whether mitochondrial stress is involved in the LPS-induced HAVIC inflammatory responses, HAVICs were treated with NAC (1 mM, Beyotime, S0077) for 1 hour prior to LPS stimulation.

To evaluate the role of IL-37 in mediating the effect of S18 on HAVICs, HAVICs were treated with IL-37 siRNA (50 nM, OBiO) for 8 hours followed by stimulation with LPS with or without S18 (0.5 *μ*M).

To determine the role of IL-37 in attenuating the mitochondrial stress in HAVICs, HAVICs were preincubated with recombinant IL-37 (0.1 ng/mL, MCE, HY-P70455) for 1 hour followed by LPS (200 ng/mL) stimulation.

### 2.4. Experimental Mouse Model

All animal experiments were performed according to the guidelines from Directive 2010/63/EU of the European Parliament on the protection of animals used for scientific purposes. The study was approved by the Ethics Committee for Animal Experiments of Southern Medical University. IL-37-Tg mice were constructed in the Shanghai Model Organisms Center. IL-37-Tg mice were constructed via PiggyBAC transposase system. Briefly, PiggyBAC mRNA was obtained by transcription in vitro. PiggyBAC mRNA and the vector containing the target insert were microinjected into the fertilized eggs of C57BL/6J mice.

Mice (8-week-old males) were separated into three groups. Mice were injected intraperitoneally with saline and fed a normal diet (*n* = 5), or mice were injected intraperitoneally with S18 (0.8 mg/kg) and fed an adenine diet (*n* = 5). As reported previously [29], 1.48 × 10^−2^ mol/kg adenine (Sigma-Aldrich, A8626) was added to the diet for 21 days. Thereafter, renal function was evaluated by examining serum BUN and creatinine levels (Mindray, China). Then, 2.27 × 10^−5^ mol/kg vitamin D (Sigma-Aldrich, C9756) dissolved in olive oil (Sigma-Aldrich, O1514) was injected intraperitoneally on 10 consecutive days. After an additional 4 days, the mice were anaesthetized by intraperitoneal injection with sodium pentobarbital, and tissue was harvested. The heart was perfused with 10 mL of normal saline under physiological pressure before tissue collection. The heart tissues were embedded in paraffin and dissected into 5 *μ*m sections. The sections were fixed in 4% paraformaldehyde for haematoxylin and eosin (H&E) staining, Von Kossa staining, and immunofluorescence staining.

### 2.5. Microscale Thermophoresis (MST)

The ability of piericidin diglycosides to bind with potential ligands was analysed using MST. The IL-37 protein (MCE, HY-P70455) was labelled with Monolith NT™ Protein Labelling Kit Blue (Nano Temper Technologies, MO-L002) according to the manufacturer's protocol. The compounds were diluted in 16 dilution steps covering the range of appropriate concentrations. After 15 minutes of incubation at room temperature, the samples were loaded into capillaries, and thermophoresis was measured on Monolith NT.115 instrument (Nano Temper Technologies, Germany). The *K*_*d*_ values were calculated using NT Analysis software (Nano Temper Technologies, Germany).

### 2.6. Molecular docking

The Schrödinger 2017-1 suite (Schrödinger Inc., New York, NY) was employed to perform the docking analysis. The IL-37 structure was retrieved from the available crystal structures (PDB: 6NCU) and constructed following the protein Preparation Wizard workflow in the Maestro package. The binding site was selected using the Grid Generation procedure. The prepared ligand was flexibly docked into the receptor using Glide (XP mode) with default parameters.

### 2.7. Statistical Analysis

Data are presented as the mean ± SEM. Statistical analyses were performed using GraphPad Prism 7.0. Comparisons between multiple groups were analysed using one-way analysis of variance (ANOVA) with a post hoc Bonferroni/Dunn test, two-group comparisons were analysed using a *t*-test, and differences were determined by the Mann–Whitney *U* test. *p* ≤ 0.05 was considered to statistical significance.

## 3. Results

### 3.1. Effects of Marine-Derived Natural Products S18 and GPA on Cell Viability

The piericidin diglycoside S18 and piericidin monoglycoside GPA were discovered in the culture broth of *Streptomyces pasmmoticus* SCSIO NS126, an actinomycete strain derived from a mangrove sediment samples that were obtained from the Pearl River estuary of the South China Sea. S18 and GPA were identified as 13-hydroxypiericidin A 10-O-*α*-D-glucose (1→6)-*β*-D-glucoside and glucopiericidin A through HRMS and NMR analyses (Figures S3 and S5), respectively, as previously reported [25]. S18, as a specific piericidin diglycoside, is a relatively rare and novel natural piericidin [23]. The chemical structures of S18 and GPA are shown in Figures 1(a) and 1(b).

HAVICs, the principal cell type of the aortic valve, exert a prominent effect on CAVD by undergoing myofibroblastic differentiation and depositing fibrotic matrix [30]. To assess the toxic effects of S18 and GPA on the proliferation of HAVICs, we treated HAVICs with different concentrations of S18 and GPA for 2 days and assessed cell viability with a Cell Counting Kit-8 (CCK-8) assay. After treatment with a series of concentrations of S18 from 0 to 4 *μ*M for 2 days, the results showed no difference in cell viability (Figures 1(c) and 1(d)). Thus, S18 has no obvious toxicity on HAVICs. However, GPA at a concentration above 0.5 *μ*M showed toxic effects on HAVICs (Figures 1(d)–1(f)).

### 3.2. S18 Suppresses LPS-Mediated Inflammatory Responses in HAVICs

To determine the role of S18 in HAVICs, we exposed cells to LPS (200 ng/mL) with increasing concentrations of S18 (0.5, 1, or 2 *μ*M) for 24 hours.  Figure 2(a) shows that S18 reduced the expression of intercellular cell adhesion molecule-1 (ICAM-1) in LPS-treated HAVICs in a dose-dependent fashion, while GPA had no effect on the level of ICAM-1 in HAVICs at the tested concentrations (Figure 2(b)). Notably, the LPS-induced increases in ICAM-1 level in HAVICs was significantly reduced by 25% with 0.5 *μ*M S18. Simultaneously, 0.5 *μ*M S18 reduced the expression of interleukin IL-8 and monocyte chemoattractant protein-1 (MCP-1) by 31% and 40%, respectively (Figures 2(c) and 2(d)). The levels of ICAM-1, IL-8, and MCP-1 genes in HAVICs were also reduced by S18 treatment (Figure 2(e)). These results demonstrate that S18 negatively regulates HAVIC inflammatory responses to LPS.

### 3.3. S18 Protects against LPS-Induced Mitochondrial Stress

Recent evidence has suggested that mitochondrial activity has a potential role in the development of cardiovascular calcification. Next, the role of S18 in mitochondrial function was explored. As expected, we found that the ROS production was upregulated 2.1 folds in LPS-treated HAVICs, while S18 treatment markedly reduced LPS-induced ROS production by over 25% (Figure 3(a)). Next, fluorescence images of JC-1 and tetramethylrhodamine, methyl ester (TMRM) staining revealed that the mitochondrial membrane potential (MMP) was upregulated by over 40% in HAVICs treated with LPS and S18, compared with that in HAVICs treated with LPS alone (Figures 3(b) and 3(c)), suggesting that S18 attenuates mitochondrial stress. Moreover, the mitochondrial quantity was determined with Mito-Tracker Green. LPS-exposed cells showed reduction in mitochondrial mass, which was indicated by the downregulation of the Mito-Tracker Green fluorescence signals. On the contrary, the LPS-induced mitochondrial dysfunction was significantly restored (approximately 40%) by S18 therapy (Figure 3(d)). Taken together, these observations reveal that LPS elicits mitochondrial dysfunction in HAVICs, which is attenuated by S18.

### 3.4. S18 Suppresses Inflammation through the NF-*κ*B p65-Dependent Pathway in HAVICs

To date, it has been well established through a variety of studies that the NF-*κ*B pathway plays an essential role in many cardiovascular diseases including CAVD, cardiac hypertrophy, and heart failure [31]. Cytokines, including ICAM-1, IL-8, and MCP-1, converge in the downstream activation of the NF-*κ*B pathway in CAVD. To investigate the mechanism by which inflammatory responses to LPS are mitigated by S18 in HAVICs, we evaluated the effect of S18 on NF-*κ*B, as it is crucial to mediate HAVIC inflammation.  Figure 4(a) shows that the induction of NF-*κ*B phosphorylation (approximately 4 folds) by LPS in HAVICs was suppressed by over 40% with S18. The immunofluorescence staining images in Figure 4(b) confirmed the inhibitory effect of S18 on LPS-induced nuclear translocation of NF-*κ*B p65 (Figure 4(b)). NAC, a classical antioxidant, has been used to scavenge ROS and prevent mitochondrial stress [32]. Next, we tested the hypothesis that the increased ROS levels induced by mitochondrial stress account for NF-*κ*B activation in HAVICs exposed to LPS. As expected, NAC treatment suppressed LPS-induced NF-*κ*B p65 phosphorylation by 25% and nuclear translocation (Figures 4(c) and 4(d)). Thus, these results suggest that S18 functions as a potent inhibitor of NF-*κ*B p65 to restrain LPS-induced inflammatory responses in HAVICs.

### 3.5. IL-37 Is Involved in the S18-Mediated Attenuation of HAVIC Inflammatory Responses to LPS

Our previous studies found that recombinant IL-37 exerts potent protective effects on CAVD and that recombinant IL-37 alleviates MyD88-mediated inflammatory mediator production after stimulating TLR2/4 in HAVICs [33]. Five patients with CAVD and four patients with non-CAVD were recruited in this study (Figure 5(a)). We also found that the level of IL-37 protein in calcified aortic valve was notably lower, compared with that in non-CAVD patients (Figures 5(a) and 5(b)). To elucidate the molecular mechanisms of S18 in HAVICs, we explored the role of IL-37 on the effect of S18-mediated attenuation of inflammatory cytokines in HAVICs. The Western blotting results showed that IL-37 was upregulated by approximately 35% in HAVICs after S18 treatment (Figure 5(c)). We also detected the expression of IL-37 in GPA-treated HAVICs. However, GPA failed to induce IL-37 expression (Figure S7). Subsequently, knockdown experiments were performed in HAVICs. As shown in Figure 5(d), the IL-37 level in HAVICs was effectively knocked down by siRNA but not by the scrambled siRNA. Moreover, the expression of ICAM-1 and IL-8 was downregulated by 25% and 20% in LPS-treated HAVICs, respectively. Thus, IL-37 knockdown significantly blunted the suppressive effect of S18 on the HAVIC inflammatory responses to LPS (Figures 5(e) and 5(f)). Collectively, it is reasonable to believe that IL-37 is a potential target of S18, but not GPA, in HAVICs.

### 3.6. IL-37 Mediates the Protection against Mitochondrial Stress in HAVICs

To investigate whether IL-37 attenuates mitochondrial stress in HAVICs, we treated HAVICs with recombinant IL-37 (0.1 ng/mL) 1 hour prior to LPS. As shown in Figures 6(a) and 6(b), recombinant IL-37 not only significantly decreased ROS levels by 30% but also increased MMP levels in HAVICs stimulated with LPS. Conversely, IL-37 knockdown through specific siRNAs further upregulated LPS-induced ROS production and decreased MMP (Figures 6(c) and 6(d)). Thus, these results suggest that downregulating IL-37 with siRNA prevents the protective effect of S18 against LPS-induced mitochondrial stress.

### 3.7. Docking Analysis of S18 and GPA with IL-37

The monomeric and dimeric forms of IL-37 have a remarkable impact on its anti-inflammatory activity. Eisenmesser et al. found that, compared with native IL-37, monomeric IL-37 shows more effective suppression of inflammatory mediators in multiple cell types [34]. To order to explore the interaction between S18 and the potential target, we selected a homology model of IL-37 (PDB code: 6NCU), which was subjected to in silico molecular docking analysis. S18 comfortably combines with the monomeric and dimeric forms of IL-37 into the binding pocket (Figure 7) with negative binding free energy values (*S* value) -6.618 and -7.042, respectively. Heparin was selected to be the positive control drug [34]. Intriguingly, heparin appeared to fit perfectly into the monomeric form of IL-37 with an *S* value of -7.290 but interacted with the dimeric form of IL-37 with an *S* value of -2.159 (Figure S8). In addition, the docking analysis of several piericidin analogues was assessed. Similar to S18, S40, a piericidin diglycoside, could be considered as a potential ligand of the IL-37 protein (Figure S8a). On the contrary, piericidin glycoside S14 and piericidin aglycone PA failed to dock with the IL-37 protein (Figure S8b-c).

As shown in Figure 7(b), S18 exhibited a vital role in the binding model, and its hydroxy groups formed hydrogen bonds with the active site residues LYS58, ARG158, and GLN160 in the monomeric form of IL-37. However, the glucoside with monosaccharides GPA (Figure 7(c)) and S14 (Figure S8b) displayed weak activity in the binding model of the monomeric form of IL-37 with S values ranging from -4 to -5, which was consistent with the corresponding MST assay results (Figure S8d). MST analysis also revealed that PA exhibited no binding activity with IL-37 (Figure S8d). Therefore, further exploration could be conducted to reveal the underlying mechanism of IL-37 that is induced by piericidin glucoside accompanied by disaccharide or monosaccharide.

### 3.8. S18 Alleviates Aortic Valve Lesions In Vivo

To further confirm the effect of S18 on CAVD, a renal dysfunction plus vitamin D-induced aortic valve calcification model was established as previously reported [29] (Figure 8(a)). IL-37 transgenic (Tg) mice were intraperitoneally injected with normal saline or S18 and fed an adenine (1.48 × 10^−2^ mol/kg) diet for 21 days to induce renal dysfunction. Other IL-37-Tg mice were intraperitoneally injected with normal saline and were fed a regular diet as a control. The levels of creatinine and blood urea (BUN) were detected (Figure S9a). Vitamin D (2.27 × 10^−5^ mol/kg) was applied to generate high calcium-induced aortic valve calcification. After vitamin D injection for 10 days, no obvious effect of vitamin D on renal function was observed (Figure S9b). After an additional 4 days of observation, the heart tissue of mice was harvested to perform H&E staining, Von Kossa staining, and immunofluorescence staining. As shown in Figure 8(b), the cardiomyocyte cross-sectional area and the aortic valve leaflet thickness were increased in the model group compared with the control group but were markedly decreased by S18 treatment. Correspondingly, the results of the Von Kossa staining illustrated that S18 impeded the aortic valve thickening and calcium deposition induced by prolonged renal dysfunction plus vitamin D administration (Figure 8(c)). In addition, immunofluorescence analysis revealed that the levels of ALP and BMP2 were increased in the thickened aortic valve tissues from the model group, but that supplemental S18 reduced the expression of ALP, and BMP2 in valve tissues (Figures 8(d) and 8(e)).

## 4. Discussion

In recent decades, valvular inflammation has been considered to occur in the initial lesions and throughout the course of CAVD [35]. Upon exposure to proinflammatory stimuli, HAVICs differentiate into osteoblast-like cells, which produce and deposit collagen matrix and bone-relaxed proteins to remodel valvular structure, resulting in valvar thickening and stiffening [11]. In this regard, investigating the molecular mechanism underlying aortic valve inflammatory responses and discovering anti-inflammatory agents may promote the development of pharmacological interventions for CAVD.

However, few studies have yet discovered novel drugs, especially marine-derived compounds, which ameliorate the inflammatory responses of HAVICs. In this study, we discovered a marine-derived piericidin diglycoside S18 with pharmacological potential and found that (1) S18 suppressed the HAVIC inflammatory responses to LPS, (2) S18 mitigated the LPS-induced mitochondrial stress implicated in HAVICs inflammation, (3) S18 interacted with IL-37 to inhibit the NF-*κ*B activation involved in the HAVIC proinflammatory pathway, and (4) administration of S18 alleviated aortic valve calcification in IL-37-Tg mice. These findings represent the therapeutic potential of S18 for CAVD and provide new insights to aid in the discovery of anti-CAVD agents from marine-derived compounds.

### 4.1. S18 Suppresses LPS-Induced Inflammation and Mitochondrial Stress in HAVICs

Haemodynamic mechanical stress and shear stress on the aortic valve damage to aortic valve endothelial cells, and then, lipoprotein (a), oxidized low-density lipoprotein (oxLDL) cholesterol, and proinflammatory factors infiltrate the valvular interstitium [36]. These factors act as damage-associated molecular patterns (DAMPs) to provoke mitochondrial stress and inflammation in AVICs [4]. Subsequently, activated HAVICs produce proinflammatory factors, including ICAM-1 [37], IL-8, and MCP-1 [38, 39], resulting in the infiltration of immune cells and a resultant further inflammatory cascade in valve tissue [39, 40]. In this regard, numerous lines of evidence indicate that valvular inflammation initiates the early stage of CAVD. Moreover, our previous studies reported that proinflammatory stimuli promote the osteogenic differentiation of HAVICs [41, 42]. Therefore, it is conceivable that agents that suppress AVIC inflammatory responses might have therapeutic potential for CAVD.

Accumulating evidence suggests that mitochondria exert a pivotal effect on the inflammatory response, and mitochondrial dysfunction is involved in numerous diseases that are characterized by chronic inflammation, including atherosclerosis, cancer, and neurodegeneration [43, 44]. Mitochondria has an important effect on cell inflammation via modulating the production of ROS and the activation of NF-*κ*B pathway. The overproduction of mitochondrial ROS and oxidative stress are the key features of mitochondrial dysfunction, which in turn leads to inflammatory responses [45]. Furthermore, inflammation induced by ROS acts as a loop, resulting in the exacerbation of tissue damage [46]. Mitochondrial dysfunction is well-known to play an essential role in the progression of atherosclerosis. Zhang et al. found that CoQ_10_ supplementation alleviates mitochondrial function, and then, the degree of atherosclerotic lesions was significantly relieved in ApoE-/- mice [47, 48]. Therefore, mitochondria are a promising therapeutic target for novel treatments of diseases with chronic inflammation.

Here, we found that S18 substantially decreased the production of ICAM-1, IL-8, MCP-1, and ROS in HAVICs treated with LPS. Additionally, S18 attenuated the LPS-induced downregulation in MMP and mitochondrial mass. These results allude to the participation of mitochondrial stress in HAVICs and demonstrate that S18 negatively regulates HAVIC inflammatory responses to proinflammatory stimuli. These findings support that S18 may have therapeutic potential for preventing aortic valve calcification.

Although CAVD is associated with various risk factors, patients with CAVD are often accompanied with diabetes or chronic kidney disease [49]. These patients have poor calcium metabolism, which results in a high calcium load and then largely contributes to the accelerated calcification of the aortic valve [50]. Thus far, no drugs have shown therapeutic effects on the initial phases of CAVD. Hence, mounting research has focused on seeking agents against CAVD. Marine-derived compounds undoubtedly have considerable potential [51]. Similarly, our in vivo studies revealed that S18 exhibited significantly alleviated aortic valve thickening, decreased calcium nodule formation, and reduced ALP and BMP2 levels in valve leaflets after prolonged exposure to renal dysfunction plus vitamin D-induced valve calcification. To the best of our knowledge, these findings represent the first report of a beneficial role of S18 on CAVD. Furthermore, the anti-inflammatory effects of S18 have clinical significance.

### 4.2. IL-37 Mediates the Protective Effects of S18 against on HAVIC Inflammatory Responses via the Inhibition of NF-*κ*B

IL-37 is a special member of the IL-1 family due to its inhibitory effects on the production of inflammatory cytokines in many kinds of cells [52]. A bulk of data corroborates the in vivo protective effect of IL-37 in disease models [53–55]. Analogously, we found that IL-37 suppresses the inflammatory and osteogenic responses to stimuli in HAVICs and ameliorates valve lesions in mice [22, 33]. In addition, as a classical inflammatory pathway mediator, NF-*κ*B is thought to induce the activation of downstream cytokines.

Given the broad therapeutic potential of IL-37 and the extensive involvement of NF-*κ*B in inflammation, we hypothesized that S18 promotes IL-37 expression to mitigate HAVIC inflammatory responses to LPS in an NF-*κ*B-dependent fashion. While verifying this hypothesis, we found that S18 upregulated the expression of IL-37 in HAVICs. Correspondingly, LPS-induced phosphorylation and nuclear translocation of NF-*κ*B p65 in HAVICs were suppressed by S18. Moreover, it is noteworthy that IL-37 appears to play a vital role in mediating the protective effects of S18 since IL-37 knockdown via siRNA blunted but did not abolish the anti-inflammatory and antioxidative effects of S18, as evidenced by the reduction but still high levels of ICAM-1 and IL-8.

Increasing evidence reveals that oxidative stress is involved in the progression of CAVD and mouse models of valve stenosis [12]. ROS has been characterized as activating proosteogenic signals and accelerating calcification of vascular smooth muscle cells in vitro [13]. However, uncertainty remains regarding the role of IL-37 in oxidative stress. Here, our pioneering study determined that IL-37 has a profound effect on oxidative stress in HAVICs. NAC inhibited inflammatory responses and NF-*κ*B phosphorylation, which suggests that oxidative stress is involved in LPS-induced inflammatory responses. We also found that S18 could not alleviate oxidative stress in the presence of IL-37 siRNA, which suggests that S18 may exert its effect on HAVICs in an IL-37-dependent manner. Accordingly, IL-37 is a key factor for the therapeutic effect of S18 on CAVD.

### 4.3. IL-37 Is a Potential Target of the Piericidin Diglycoside S18 in HAVICs

To date, compounds that inhibit or activate the IL-37 protein to achieve therapeutic effects remain to be discovered. A total of 5 piericidin compounds were applied to the docking analysis, consisting of the aglycone PA, the piericidin diglycosides S18 and S40, and the piericidin monoglycosides GPA and S14. MST and docking analysis provided direct evidence that the piericidin diglycosides S18 and S40 may be potential candidates that bind to and activate the IL-37 protein. In contrast, the piericidin monoglycosides, GPA and S14, exerted no IL-37-binding activity. Moreover, the toxicity of S18 is less than that of GPA in HAVICs. In these contexts, compared to piericidin monoglycoside, piericidin diglycosides have a greater therapeutic potential for CAVD.

Agents with excellent pharmacological activity for CAVD are expected to be discovered. Numerous studies have been performed to discover novel drugs from a variety of natural products [56, 57]. Notably, marine natural products represent the most abundant source of novel compounds that maybe overcome the limitations of other anti-CAVD drug discovery approaches and become pioneering agents in the treatment of CAVD. Additionally, further exploration of the effect of these drugs on CAVD will not only have crucial complications for the understanding of cardiovascular diseases but also provide a rationale for discovering new therapeutic strategies.

There are several limitations in this study. First, the direct detection of the expression of IL-37 in animal experiments is impossible, because mice do not have a homologue gene for human IL-37. Therefore, IL-37-Tg mice were used to examine the effect of S18 in vivo. Second, hyperlipidaemia and osteoblast-like differentiation contribute to the progression of CAVD. The effects of S18 on osteogenic responses and hyperlipidaemia should be further examined. Future studies should explore the anti-CAVD mechanism of S18.

## 5. Conclusion

In conclusion, this study demonstrates that S18 attenuates HAVIC inflammatory responses in vitro and alleviates mouse aortic valve lesions in vivo. S18 promotes and interacts with IL-37 to inhibit mitochondrial stress and NF-*κ*B activation which is responsible for the anti-CAVD effect of S18. Moreover, the piericidin diglycoside S18 directly combined with IL-37 protein, while monoglycosides exerted no IL-37-binding activity. Overall, our findings provide a novel potential treatment for preventing the progression of valvular calcification.

## Figures and Tables

**Figure 1:** Viability of HAVICs following S18 and GPA treatment. (a, b) The structure of S18 and GPA. (c–f) Cell viability with or without S18 or GPA treatment for 2 days, *n* = 5. ^∗^*p* < 0.05 compared with the control.

**Figure 2:** S18 ameliorates inflammatory responses in vitro. (a, b) Cells were stimulated with 200 ng/mL LPS and then treated or not treated with S18 and GPA for 24 hours. Immunoblotting results show the expression of ICAM-1 in HAVICs, *n* = 4. (c) The expression of ICAM-1, IL-8, and MCP-1 was determined via Western blotting and quantification analysis after 24 hours of treatment with S18 (0.5 *μ*M), *n* = 5. (d) The levels of IL-8 and MCP-1 in the culture medium of cells from valves were tested by enzyme-linked immunosorbent assay (ELISA), *n* = 5. (e) The mRNA levels of ICAM-1, IL-8, and MCP-1 were determined by quantitative real-time polymerase chain reaction (qRT-PCR), *n* = 5. Error bars represent the mean ± SEM, ^#^*p* < 0.05, ^##^*p* < 0.01, and ^###^*p* < 0.0001 vs. control; ^∗^*p* < 0.05, and ^∗∗^*p* < 0.01 vs. the LPS group.

**Figure 3:** S18 prevents LPS-induced mitochondrial dysfunction in HAVICs. Cells were treated with LPS (200 ng/mL) in the presence or absence of S18 for 24 hours. (a) Fluorescence images show the production of ROS in HAVICs using the 2,7-dichlorodihydrofluorescein diacetate (DCFH-DA) fluorescent dye, *n* = 5. Scale bar = 100 *μ*m. (b) Fluorescence images of HAVICs stained with TMRM, *n* = 5. Scale bar = 25 *μ*m. (c) The MMP was detected with JC-1 staining in HAVICs, *n* = 5. Scale bar = 100 *μ*m. (d) Fluorescence intensity of Mito-Tracker Green staining is shown in HAVICs, *n* = 5. Scale bar = 100 *μ*m. The data are shown as the mean ± SEM. ^#^*p* < 0.05 vs. control; ^∗^*p* < 0.05 vs. the LPS group.

**Figure 4:** S18 prevents the activation of NF-*κ*B p65 against inflammation. HAVICs were treated with LPS (200 ng/mL) for 4 hours in the presence or absence of S18. (a) Western blot analysis shows that S18 reduced the phosphorylation of NF-*κ*B p65 in HAVICs, *n* = 5. (b) Representative images show intranuclear localization of NF-*κ*B p65 in HAVICs stimulated with LPS and extranuclear localization of NF-*κ*B p65 after HAVICs were treated with S18. Scale bar = 50 *μ*m. (c, d) Data show that NAC treatment reduces NF-*κ*B phosphorylation in HAVICs, *n* = 4. Images show that NAC treatment attenuates LPS-induced intranuclear localization of NF-*κ*B p65 in HAVICs. Scale bar = 50 *μ* m. Data are shown as the mean ± SEM. ^#^*p* < 0.05, and ^##^*p* < 0.01 vs. control; ^∗^*p* < 0.05 vs. LPS alone.

**Figure 5:** IL-37 activation is required for the downregulation of inflammatory cytokines caused by S18. (a, b) HE staining of aortic valve from patients with CAVD or non-CAVD patients, and the expression of IL-37 in valve tissue was detected by immunofluorescent staining. ^∗∗^*p* < 0.01 compared with the non-CAVD group, scale bar = 50 *μ*m, *n* = 4. (c, d) Representative immunoblots and the corresponding quantification of IL-37 in HAVICs, *n* = 5. ^∗^*p* < 0.05 compared with the LPS group. (e, f) Representative immunoblots and ELISA showing the protein expression of ICAM-1 and IL-8 in LPS and S18-treated HAVICs in combination with IL-37 knockdown. Cells with scrambled siRNA were used as controls, *n* = 4. Data are shown as the mean ± SEM. ^∗∗^*p* < 0.01, and ^∗^*p* < 0.05.

**Figure 6:** S18 prevents against mitochondrial dysfunction in an IL-37-dependent manner. HAVICs were treated with LPS (200 ng/mL) in the presence or absence of IL-37 (0.1 ng/mL) for 24 hours. (a) Fluorescence images with DCFH-DA dye show the ROS production, *n* = 4. Scale bar = 100 *μ*m. (b) Fluorescence images of HAVICs stained with TMRM, *n* = 4. Scale bar = 50 *μ*m. Cells were treated with IL-37 siRNA (50 nM, OBiO) following stimulation with LPS (200 ng/mL) with or without S18 (0.5 *μ*M). (c) Fluorescence images using DCFH-DA fluorescent dye show ROS production, *n* = 4. Scale bar = 100 *μ*m. (d) Fluorescence intensity of TMRM staining is shown, *n* = 4. Scale bar = 50 *μ*m. Data are shown as the mean ± SEM. ^#^*p* < 0.05 compared with the control group, ^∗^*p* < 0.05.

**Figure 7:** S18 directly binds the monomeric forms of IL-37 (6NCU). The detailed docking mode of (a) heparin/IL-37, (b) S18/IL-37, and (c) GPA/IL-37 with docking pock. The affinity of (d) heparin/IL-37 (*K*_*d*_ = 36.0 *μ*M), (e) S18/IL-37 (*K*_*d*_ = 84.2 *μ*M), and GPA/IL-37 (*K*_*d*_ = no binding) binding as analysed by MST assay. Data are shown as the mean ± SEM, *n* = 3.

**Figure 8:** Evaluation of the therapeutic efficacy of S18 in IL-37-Tg mice. (a) Timeline diagram of S18 administration in the aortic valve calcification model. (b) Pathological changes in cardiomyocytes and aortic valves in the aortic valve calcification model. HE staining of cardiomyocytes and aortic valves. Scale bar = 200 *μ*m. (c) Von Kossa staining in the aortic valve calcification model. Scale bar = 50 *μ*m. (d, e) Representative immunofluorescence images in mouse aortic valves. Scale bar = 50 *μ*m, *n* = 5. Data are the mean ± SEM. ^##^*p* < 0.01 vs. sham; ^∗∗^*p* < 0.01 vs. the Vit D group.

## Data Availability

The data used to support the findings of this study are included within the article.

## Abbreviations

AVICs: Interstitial cells of aortic valve cells
CAVD: Calcific aortic valve disease
CKD: Chronic kidney disease
DAMPs: Damage-associated molecular patterns
DCFH: 2,7-Dichlorodihydrofluorescein diacetate
ELISA: Enzyme-linked immunosorbent assay
H&E: Hematoxylin and eosin
HPLC: High-performance liquid chromatography
HRMS: High-resolution mass spectrometry
HAVICs: Human interstitial cells of aortic valve cells
ICAM-1: Intercellular cell adhesion molecule-1
IL-37: Interleukin-37
BUN: Blood urea
IL-37-Tg mice: IL-37 transgenic mice
IL-8: Interleukin-8
LC-MS/MS: Liquid chromatography-tandem mass spectrometry
LPS: Lipopolysaccharide
MCP-1: Monocyte chemoattractant protein-1
MMP: Mitochondrial membrane potential
MST: Microscale thermophoresis
NAC: N-acetyl-L-cysteine
NMR: Nuclear magnetic resonance
oxLDL: Oxidized low-density lipoprotein
qRT-PCR: Quantitative real-time polymerase chain reaction
ROS: Reactive oxygen species
siRNA: Small interfering RNA
TLR4: Toll-like receptor 4
TMRM: Tetramethylrhodamine, ethyl ester.

## Supplementary Materials

Supplementary Materials Supplementary materials and methods: additional figures illustrating structure elucidation and spectral data of S18, GPA, S40, S14, and PA, as well as their spectra (IR, MS, and NMR) (Figure S1-S6); the effect of GPA on expression of IL-37 protein (Figure S7); the structures of piericidin analogues subjected to the docking analysis, the docking results of some piericidin aglycones binding with IL-37 (6NCU) (Figures S8); renal function in mice (Figure S9); demographic characteristic of enrolled patients (Table S1); the primer information (Table S2).
